The article "CT Image Feature under Intelligent Algorithm in the Evaluation of Continuous Blood Purification in the Treatment and Nursing of Pulmonary Infection-Caused Severe Sepsis" was retracted in 2023. Reasons: signs of a paper mill; suspected computer-generated content; unreliable results or conclusions; concerns about the data.

# CT Image Feature under Intelligent Algorithm in the Evaluation of Continuous Blood Purification in the Treatment and Nursing of Pulmonary Infection-Caused Severe Sepsis

**DOI:** 10.1155/2021/2281327

**Published:** 2021-11-28

**Authors:** Liping Liu, Yanyan Liu, Aimin Xing, Siyu Chen, Mingli Gu

**Affiliations:** Department of Critical Care Medicine, Affiliated Hongqi Hospital of Mudanjiang Medical University, Mudanjiang, 157011 Heilongjiang, China

## Abstract

This study was to explore the CT image features based on intelligent algorithm to evaluate continuous blood purification in the treatment of severe sepsis caused by pulmonary infection and nursing. 50 patients in the hospital were selected as the research objects. Convolutional neural network algorithm was used to segment CT images of severe sepsis caused by pulmonary infection. They were randomly divided into 25 cases of experimental group and 25 cases of control group. The experimental group was given continuous blood purification treatment, combined with comprehensive nursing. The control group was given routine treatment and basic nursing. Fasting plasma glucose (FPG) and fasting insulin (FIN), interleukin-6 (IL-6), tumor necrosis factor (TNF-*α*), high-sensitivity c-reactive protein (hs-CRP) levels, CD_3_^+^, CD_4_^+^, CD_4_^+/^CD_8_^+^ levels, ICU monitoring time, malnutrition inflammation score (MIS), and incidence of adverse events were compared between the two groups before and after treatment. There was no difference in FPG and FIN between the two groups before treatment. After treatment, the FPG and FIN of the experimental group were lower than those of the control group, and there was statistical significance (*P* < 0.05). There was no difference in IL-6, TNF-*α*, and hs-CRP between the two groups before treatment. After treatment, IL-6, TNF-*α*, and hs-CRP in the experimental group were lower than those in the control group. There was no difference in the percentage of CD_3_^+^, CD_4_^+^, and CD_4_^+/^CD_8_^+^ between the two groups before treatment. After treatment, the CD_3_^+^, CD_4_^+^, and CD_4_^+^/CD_8_^+^ in the experimental group were higher than those in the control group. The ICU monitoring time, MIS, and incidence of adverse events in the experimental group were lower than those in the control group (*P* > 0.05). Convolutional neural network algorithm can accurately identify and segment CT images of patients with severe sepsis, which has high clinical application value. Continuous blood purification therapy can effectively control blood glucose level, improve immune function, and reduce the content of inflammatory factors in patients with severe sepsis caused by pulmonary infection. Effective nursing measures can improve the therapeutic effect.

## 1. Introduction

Sepsis refers to a systemic inflammatory syndrome caused by the imbalance of human response to infection, which can be life threatening and lead to systemic organ dysfunction [1]. According to a statistical report on sepsis, about 30 million people die of severe sepsis every year in the world, with a mortality rate of 50%, which has seriously threatened human life [2, 3]. There are many factors leading to sepsis, mainly because the immune system and inflammatory reaction of the body are infected by serious pathogens and enter the blood through inflammatory pus, resulting in serious bacterial infection in the blood system, leading to coagulation disorder, multiple organ failure, and infection in various parts of the body, such as lung infection [4, 5]. According to the severity of sepsis, sepsis can be divided into three stages: sepsis, severe sepsis, and septic shock [6, 7]. Because the onset of sepsis is urgent and dangerous, the stage from sepsis to severe sepsis is fast, and the time from severe sepsis to septic shock is very short, which takes less than a day. Therefore, it is very necessary to determine the location of focus and complications of severe sepsis as soon as possible to guide doctors to formulate effective treatment plans. However, CT images often used in clinic need imaging doctors to manually divide and process the image. Manual segmentation is highly subjective only by relying on the imaging doctors' many years of clinical experience and professional knowledge. If the patient has more imaging data, it is not only time-consuming but also cannot effectively ensure high-quality results. Therefore, there is an urgent need for an alternative artificial intelligence algorithm to complete lesion division. Convolution neural network algorithm is a new intelligent algorithm in recent years. It can divide medical image images efficiently and quickly, with an average time of 0.9 s [8]. Therefore, it has attracted much attention in medical assisted division of lesion sites. Convolution neural network algorithm is an automatic intelligent algorithm based on computer technology and mathematical data processing. It can extract the features of the region of interest of medical image without human intervention, then classify the features, and finally output the target data [9]. In some studies, the convolution neural network algorithm is used to segment the cardiac CT image, locate the target area, intercept the cardiac image through the obtained characteristic image, and compare the segmentation results with other algorithms. It is found that the convolution neural network algorithm can fully meet the requirements of fully automatic segmentation of cardiac CT image. Moreover, the segmented image results are more helpful for clinicians to accurately obtain the patient's heart contour [10]. At present, there is little research on the application of convolutional neural network algorithm in CT images of patients with severe sepsis. Therefore, in this study, the convolutional neural network algorithm was used to segment the CT images of patients with pulmonary infection to severe sepsis in order to assist clinicians in the early diagnosis of severe sepsis.

The pathogenesis of sepsis is complex, and the clinical manifestations lack obvious specificity. Therefore, for patients with no obvious clinical symptoms, laboratory examinations such as blood, biochemistry, and microorganism are regarded as the main diagnostic means [11–13]. Conventional laboratory tests such as leukocyte count can no longer meet the early diagnosis of severe sepsis and the judgment of the development stage of the disease. Therefore, more and more scholars will start to monitor the factors causing sepsis, such as the expression of inflammatory factors, genes involved in apoptosis, proteins, and other biomarkers related to severe sepsis. Studies found that during the onset of sepsis, because the immune system is constantly stimulated by inflammatory factors, the body's inflammatory response is out of control, and the immune system secretes many inflammatory mediators, such as interleukin-6 (IL-6), high-sensitivity c-reactive protein (hs-CRP), and tumor necrosis factor (TNF-*α*). It accelerates the decomposition rate of protein in muscle so that serum albumin cannot be effectively synthesized, resulting in hypoproteinemia [14, 15]. If the inflammatory reaction cannot be prevented in time, the severe sepsis is not only easy to be aggravated but also has many serious adverse complications, such as shock, low blood pressure, and multiple organ failure [16–18]. Therefore, it is of great significance to monitor the immune system in patients with severe sepsis.

For the treatment of sepsis, conventional sepsis diagnosis and treatment guidelines cannot achieve ideal therapeutic effect. Continuous blood purification treatment can effectively remove inflammatory mediators and toxic substances and improve immune disorders by inputting replacement fluid. Moreover, the nursing of patients with severe sepsis is also one of the important links to ensure continuous blood purification treatment [19, 20]. There are many literature reports on the treatment of sepsis, but there are few relevant data on the treatment and nursing of severe sepsis caused by pulmonary infection. Therefore, in this study, different intervention methods were performed for patients with severe sepsis caused by pulmonary infection, and various indicators before and after treatment were compared to explore the clinical efficacy of continuous blood purification treatment in severe sepsis and the application of nursing, providing a reference basis for clinical treatment of patients with severe sepsis caused by pulmonary infection.

## 2. Methods

### 2.1. Research Objects

Fifty patients admitted to the hospital from May 2019 to June 2021 were selected as the research objects. There were 29 male patients and 21 female patients. Their ages ranged from 40 to 79, with a mean age of 59.5 years. The patients were randomly divided into 25 cases of experimental group and 25 cases of control group. Patients in the experimental group were given continuous blood purification treatment and integrated nursing based on conventional treatment. Patients in the control group were given routine treatment and basic nursing. All patients and their families in this study signed an informed consent, and the study was approved by the Ethics Committee of Hospital.

Inclusion criteria are as follows: (i) patients are aged between 40 and 79; (ii) the patient's condition according to the sepsis diagnostic criteria formulated by the American Thoracic Society and the European Society of Intensive Care Medicine, it was confirmed that the diagnosis result was severe sepsis caused by pulmonary infection; (iii) all clinical information of patients is complete; (iv) all patients had no other pulmonary complications, such as lung tumors; (v) the patient had no history of taking immunosuppressive drugs.

Exclusion criteria are as follows: (i) age inconsistency, (ii) severe coagulation disorders or diseases of the blood system, (iii) have a history of diabetes, and (iv) mental problems or consciousness disorders, poor compliance.

### 2.2. CT Imaging Scanning

The scanning equipment adopts 64 row spiral CT scanner for enhanced scanning. The scanning layer thickness was 4.5 mm, the layer spacing was 0.8 mm, the contrast agent was Ultravist, and the dose was 50 mL. The pulmonary CT findings of all patients were observed.

### 2.3. Segmentation of Lesion Location by Convolution Neural Network Algorithm

Convolution neural network algorithm is evolved from biological concept and belongs to deep feedback artificial neural network. It was first used to simulate the visual behavior of human cerebral cortex and then gradually applied to computer feature extraction to realize the nonlinear representation of the input data.

Generally, the classical convolution neural network algorithm structure includes several network data layers, such as input layer, convolution layer, pooling layer, activation layer, full connection layer, and output layer. Different network layers have different ways to process data, but they will eventually combine to complete a whole image recognition and segmentation process. The convolution neural network layers are connected with each other through corresponding neural nodes. By inputting information from the input layer and entering a series of convolution operations and pooling operations, the characteristic signals of the original data can be extracted and classified and mapped to the full connection layer by using the activation function [9, 21]. In view of the fact that the convolution neural network algorithm can extract and classify the features of the original data, this study uses this algorithm to segment the CT scan images of patients with severe sepsis caused by lung infection, in order to provide reference for rapid and efficient clinical diagnosis of severe sepsis. Taking segmented lung image as an example, Figure 1 shows the basic structure of convolutional neural network algorithm.

### 2.4. Image Segmentation Evaluation Index

In order to quantitatively evaluate the segmentation results of CT images of severe sepsis caused by lung infection, the segmentation performance of convolutional neural network algorithm will be measured by three indexes: segmentation accuracy, specificity, and sensitivity. This study is compared with the QTSU algorithm [22]. For the segmentation result of the algorithm, the accuracy indicates that the segmentation result is the proportion of the real lesion area in the real result. The larger its value, the more suitable the algorithm for the image segmentation. The three indicators are defined as follows.

(1) $$\begin{array}{c} \text{Accuracy}=\frac{\text{TP}+\text{TN}}{\text{TP}+\text{FP}+\text{TN}+\text{FN}}, \end{array}$$

(2) $$\begin{array}{c} \text{Specificity}=\frac{\text{TN}}{\text{TN}+\text{FP}}, \end{array}$$

(3) $$\begin{array}{c} \text{Sensitivity}=\frac{\text{TP}}{\text{TP}+\text{FN}}. \end{array}$$

Among them, TP indicates that the segmentation algorithm is the same as the real result, which is the real lesion area. TN indicates that the segmentation result of the algorithm is the same as the true result, and there is no lesion. FP indicates that the segmentation result of the algorithm is the real lesion area, and the real result has no lesion. FN indicates that the segmentation result of the algorithm is no lesion, and the real result has lesion.

### 2.5. Treatment Methods

The patients in the control group received routine treatment. The treatment plan referred to the routine treatment in the 2020 *Sepsis Treatment Guide*, and the patients were given routine care during the treatment. The patient's blood pressure, pulse, monitoring time, mechanical ventilation time, and mortality were monitored.

The patients in the experimental group were treated with continuous blood purification based on routine treatment. The treatment equipment is German Gambro Lundia blood purifier. The continuous vein-vein hemodialysis filtration mode was applied, the blood flow velocity was set to 150-180 mL/h, and the ultrafiltration volume was adjusted according to the patient's volume load. Unfractionated heparin was used in anticoagulant therapy. Each treatment lasted for at least 12 hours for one week. On this basis, psychological, anticoagulant care, and nutritional support nursing were given to the patients in the experimental group.

### 2.6. Observation Indicators

Fasting plasma glucose (FPG) and fasting insulin (FIN) were compared between the two groups before and after treatment. The changes of serum inflammatory factors before and after treatment were compared between the two groups: IL-6, TNF-*α*, and hs-CRP. The changes of T lymphocyte subsets including CD_3_^+^, CD_4_^+^, and CD_8_^+^ were compared between the two groups. The ICU monitoring time of the two groups was compared; the higher the specified score of malnutrition inflammation score (MIS) after one week of treatment, the more serious the malnutrition and inflammation of the patients, with the highest score of 20 points and the occurrence of adverse events (this study specifically refers to coagulation, bleeding, and extubation during cardiopulmonary bypass).

### 2.7. Statistical Analysis

All data were analyzed by SPSS 20.0 statistical software. The measurement data were expressed in the form of mean ± standard deviation by *t-*test, and the counting data were measured by *χ*^2^ test. When *P* < 0.05, the difference was statistically significant.

## 3. Results

### 3.1. Segmentation Results of Convolution Neural Algorithm

The CT images of patients with severe sepsis caused by pulmonary infection were divided by convolution neural network algorithm. The results are illustrated in Figure 2. Compared with the CT image segmentation results of sepsis patients by the QTSU algorithm, the convolution neural network algorithm used in this study has more accurate range, clearer boundary, and higher image quality. The lesion site is marked in green. Through the quantitative analysis of three indexes, the accuracy, specificity, and sensitivity of the algorithm used in this study are 94.23%, 94.41%, and 93.28%, which are higher than those of the QTSU algorithm, and the difference is significant (*P* < 0.05) (Figure 3). It shows that the convolution neural network algorithm can effectively realize the accurate segmentation of imaging images of patients with sepsis, and the segmentation quality is good, which can assist doctors in the diagnosis of severe sepsis.

### 3.2. Basic Data of Two Groups of Patients

A total of 50 patients were randomly divided into 25 cases in the experimental group and 25 cases in the control group. There was no significant difference between the two groups (*P* > 0.05) (Table 1).

### 3.3. Comparison Results of FPG and FIN between the Two Groups before and after Treatment

The blood glucose levels of the two groups before and after treatment are shown in Figure 4. FPG and FIN decreased in both groups before and after treatment. Compared with the control group, the decline degree of the two indexes in the experimental group was greater. There was no difference between the two groups before treatment. After treatment, FPG was 7.31 ± 1.64 and FIN was 16.12 ± 1.92 in the control group, and FPG was 6.37 ± 1.52 and FIN was 13.84 ± 1.86 in the experimental group, which were higher in the experimental group than those in the control group, and the difference between the two groups was statistically significant (*P* < 0.05).

### 3.4. Changes of Inflammatory Factors in the Two Groups before and after Treatment

The changes of inflammatory factors in the two groups before and after treatment are shown in Figure 5. The content of serum inflammatory factors decreased in both groups before and after treatment. There was no difference between the two groups before treatment. After treatment, IL-6 was 125.81 ± 14.24, TNF-*α* was 51.34 ± 6.47, and hs-CRP was 1.26 ± 0.37 in the experimental group, which were lower than 139.63 ± 16.63, 69.45 ± 7.56, and 1.58 ± 0.21 in the control group, with statistical significance (*P* < 0.05). The content of three inflammatory factors in the experimental group was lower than that in the control group.

### 3.5. Changes of T Cell Subsets in the Two Groups before and after Treatment

The changes of T cell subsets in the two groups before and after treatment are illustrated in Figure 6. The indexes before treatment were significantly different. After treatment, the percentages of CD_3_^+^ and CD_4_^+^ increased significantly, while the percentages of CD_8_^+^ decreased significantly (*P* < 0.05).

### 3.6. Nursing-Related Index Results of Two Groups of Patients

In this study, ICU monitoring time, MIS after one week of treatment, and the occurrence of adverse events (this study specifically refers to coagulation, bleeding, and extubation during cardiopulmonary bypass) were used to evaluate the impact of continuous bleeding purification treatment on nursing in the treatment process. The nursing-related index results of the two groups are illustrated in Figure 7. ICU monitoring time, MIS, and adverse events in the experimental group were lower than those in the control group. The incidence of adverse events was 16% (4/25) in the experimental group and 32% (8/25) in the control group. Compared with the control group, the incidence of adverse events in the experimental group was smaller.

## 4. Discussion

Sepsis is a systemic inflammatory runaway reaction after the body is infected by pathogenic microorganisms. The inflammatory reaction further leads to multiple organ dysfunction, which will seriously develop into septic shock [1]. Sepsis is often caused by severe trauma, burns, major surgical bleeding, serious infection of various organs, and other factors. The common type of sepsis in clinic is severe sepsis caused by pulmonary infection. The high mortality rate lies in the acute onset of sepsis and the dangerous course of disease.

However, because severe sepsis has no specific clinical symptoms, it can only be judged from imaging, biochemical indexes, microorganisms, and other laboratory tests. Therefore, rapid and accurate identification of imaging lesions of sepsis is of great significance for early diagnosis. With the development of computer technology, convolution neural network algorithm is gradually widely used in medical image recognition and lesion division. In this study, the convolution neural network algorithm is used to segment the CT images of patients with severe sepsis caused by pulmonary infection. The results show that compared with other algorithms, the image quality of the algorithm used in this paper is higher, the accuracy is higher than the index value of the QTSU algorithm, and the difference is significant (*P* < 0.05). It is suggested that the convolution neural network algorithm can effectively realize the accurate segmentation of imaging images of patients with sepsis, and the segmentation quality is good, which can assist doctors in the diagnosis of severe sepsis. This is consistent with the reported results [23].

At present, the clinical treatment of severe sepsis caused by pulmonary infection is mainly continuous blood purification. However, due to the complex pathogenesis of sepsis, which involves multiple tissues and organs of the body, patients with severe sepsis will have a rapid increase in blood glucose level. After being affected by infectious stress factors, the body has its own mechanism of adaptation, that is, insulin resistance and secondary hyperglycemia. However, this protective mechanism will not only inhibit the regeneration of liver glycogen by insulin in vivo but also weaken the ability of glucose treatment. Therefore, the blood glucose level and insulin in patients with severe sepsis will be greatly affected [24]. This study found that the FPG and FIN of the experimental group after continuous blood purification treatment were lower than those of the control group. It is consistent with the published research results [25]. In addition, uncontrolled inflammatory response is also considered to be an important basis for the pathogenesis of sepsis. Lymphocytes in patients with severe sepsis will undergo much apoptosis, which will promote the intensification of inflammatory response and immune dysfunction. Studies have shown that inflammatory factors such as serum TNF-*α*, IL-6, and hs-CRP and the percentages of CD_3_^+^, CD_4_^+^, and CD_4_^+^/CD_8_^+^ related to immune function have changed significantly after blood purification treatment, indicating that continuous blood purification treatment can significantly reduce the inflammatory state [26, 27]. The results of this study are consistent with the report. This study also found that in the treatment process of continuous blood purification, the comprehensive nursing of patients with severe sepsis can effectively shorten the ICU monitoring time, reduce the incidence of adverse events, and improve malnutrition inflammation.

## 5. Conclusion

Convolution neural network algorithm can accurately identify and segment CT images of patients with severe sepsis, which has high clinical application value. Continuous blood purification treatment for patients with severe sepsis caused by pulmonary infection can effectively control blood glucose level, improve immune function, and reduce the content of inflammatory factors. Effective nursing measures can improve the treatment effect. However, there are still some shortcomings in this study. The sample size collected is small, and more sample studies need to be carried out in the future to obtain more detailed results.

## Figures and Tables

**Figure 1:** Algorithm structure of convolutional neural network.

**Figure 2:** CT image segmentation results of sepsis patients with different algorithms. (a) The original CT image of sepsis patients caused by pulmonary infection. (b) The results of lesion segmentation using the QTSU algorithm. (c) The results of lesion segmentation using convolution neural network algorithm.

**Figure 3:** Index comparison of different algorithms. (a) The accuracy comparison results between different algorithms. (b) The specificity comparison results between different algorithms. (c) The sensitivity comparison results between different algorithms.

**Figure 4:** Comparison of blood glucose levels between the two groups before and after treatment. (a) The FPG level before and after treatment. (b) The FIN level before and after treatment. ^∗^*P* < 0.05, with statistical significance.

**Figure 5:** Comparison of inflammatory factors between the two groups before and after treatment. (a) The level of IL-6 before and after treatment. (b) The level of TNF-*α* before and after treatment. (c) The comparison of hs-CRP before and after treatment. ^∗^*P* < 0.05, with statistical significance.

**Figure 6:** Changes of indexes related to immune function in the two groups before and after treatment. (a) The changes of CD_3_^+^ in the two groups before and after treatment. (b) The changes of CD_4_^+^ in the two groups before and after treatment. (c) The changes of CD_4_^+^/CD_8_^+^ levels in the two groups before and after treatment. ^∗^*P* < 0.05, with statistical significance.

**Figure 7:** Nursing-related comparison of two groups of patients during treatment. (a) ICU monitoring time comparison results. (b) MIS comparison results. (c) The comparison results of adverse events between the two groups. ^∗^*P* < 0.05, with statistical significance.

**Table 1:** Basic data of two groups of patients.

Group	Age	Gender (men/women)	BMI (kg/m^2^)	Primary disease
Test group (*n* = 25)	60.7 ± 5.3	17/10	25.8 ± 4.2	16
Control group (*n* = 25)	59.8 ± 8.7	12/11	24.3 ± 3.6	13
*P*	0.764	0.593	0.624	0.856

## Data Availability

The data used to support the findings of this study are available from the corresponding author upon request.
